RETRACTED

# Dielectrophoresis-Based Method for Measuring the Multiangle Mechanical Properties of Biological Cells

**DOI:** 10.1155/2020/5358181

**Published:** 2020-04-06

**Authors:** Botao Zhu, Wanting Li, Mingjie Zhu, Po-Lin Hsu, Lining Sun, Hao Yang

**Affiliations:** ^1^Robotics and Microsystems Center, School of Mechanical and Electric Engineering, Soochow University, Suzhou, Jiangsu, China; ^2^Artificial Organ Technology Laboratory, School of Mechanical and Electric Engineering, Soochow University, Suzhou, Jiangsu, China

## Abstract

The mechanical properties of cells are closely related to their physiological functions and states. Analyzing and measuring these properties are beneficial to understanding cell mechanisms. However, most measurement methods only involve the unidirectional analysis of cellular mechanical properties and thus result in the incomplete measurement of these properties. In this study, a microfluidic platform was established, and an innovative microfluidic chip was designed to measure the multiangle cellular mechanical properties by using dielectrophoresis (DEP) force. Three unsymmetrical indium tin oxide (ITO) microelectrodes were designed and combined with the microfluidic chip, which were utilized to generate DEP force and stretch cell from different angles. A series of experiments was performed to measure and analyze the multiangle mechanical properties of red blood cells of mice. This work provided a new tool for the comprehensive and accurate measurement of multiangle cellular mechanical properties. The results may contribute to the exploration of the internal physiological structures of cells and the building of accurate cell models.

## 1. Introduction

The mechanical properties of cells affect cellular growth, differentiation, division, and apoptosis [1, 2]. Changes in these properties are the external manifestations of a decline in cell physiological functions; this decline eventually leads to various diseases [3–5]. Numerous advanced technologies and equipment, such as atomic force microscope, microinjection, micropipette, and optical tweezers, are used to measure cellular mechanical properties [1, 6–9]. Among these methods, devices and equipment are in direct contact with cells, which may cause damage. Dielectrophoresis (DEP) has attracted increasing attention because of its advantages, such as label-free, low cost, high throughput, and minimal damage [10, 11].

In many experiments that use DEP to measure the cellular mechanical properties, precious metal electrodes, such as gold and platinum, require magnetron sputtering, which is complex and expensive. Indium tin oxide (ITO) electrodes have low cost and are simple to manufacture and thus widely used in measuring the mechanical properties of cells, such as red blood cells and NB_4_ [12–14]. However, the majority of previous studies only performed a unidirectional measurement of the cellular mechanical properties and therefore resulted in incomprehensive measured data. In addition, the cytoplasm and nucleus are not completely symmetrical because of the nonuniformity of the physiological structures of the cells [15–17], and cellular mechanical properties in different directions may be inconsistent. Measuring the multiangle cellular mechanical properties can provide comprehensive and accurate data, and this process is convenient for studying the physiological structures of cells and building cell models. Therefore, a method that can quickly and accurately measure multiangle cellular mechanical properties must be developed.

RETRACTED

In this study, an innovative platform based on the principle of DEP that can measure the multiangle mechanical properties of cells was built. This platform mainly included a microscope, a voltage signal generator, two microfluidic pumps, and a microfluidic chip. The microfluidic chip contained three ITO electrodes to form nonuniform electric fields in different directions for the measurement of multiangle cellular mechanical properties. A series of experiments were performed to stretch the red blood cells of mice by using ITO electrodes. The analytical results showed that the mechanical properties of the red blood cell were almost the same in different directions. The proposed method also provides a new technique for studying the cellular mechanisms at the single-cell level, which helps to explore the internal physiological structure of cells. The designed microfluidic chip increases the DEP force (resultant force) at low voltages, thereby reducing damage in cells and increasing the efficiency of cell manipulation processes, such as cell rotation, separation, and transportation.

## 2. Materials and Methods

### 2.1. Sample Preparation

Blood samples were collected from the veins of healthy mice, and ethylenediaminetetraacetic acid anticoagulant was added to the samples to prevent blood clotting. Then, the samples were stored in a sterile environment at 4°C before the experiment. Appropriate amounts of red blood cells were added to the DEP buffer, which contained 8.5% *w*/*w* sucrose, 0.3% *w*/*w* glucose, and 20 mg/L CaCl_2_. The electrical conductivity and relative permittivity were 10 mS/m and 78, respectively [18, 19]. Prior to the experiment, the microchannels were rinsed with deionized water and absolute ethanol and treated with 1% BSA to prevent cell adhesion. Experiments were completed within 2 h for the maintenance of cell viability.

RETRACTED

### 2.2. Design and Manufacture of Microfluidic Chip

The microfluidic chip can be divided into two functional regions, namely, the cell focusing and stretching regions (Figure 1). Three inlets were designed in the cell focusing region. The middle microchannel was the cell injection microchannel, while the other two microchannels on both sides were used to inject the DEP buffer. The cell microchannel has a height of 50 *μ*m, a width of 600 *μ*m, and a length of 3 cm. The buffer microchannel has a height of 50 *μ*m, a width of 200 *μ*m, and a length of 600 *μ*m. The appropriate flow rate was adjusted. The cells were made to continuously flow in the middle of the microchannel because of the laminar flow, which facilitated a more efficient capture of the cells at the edge of the ITO electrodes. The cell stretching region mainly included three ITO electrodes, in which sine wave signals were applied in different ways between the three ITO electrodes to generate a multidirectional DEP force to measure and analyze the multiangle cellular mechanical properties.

The manufacture of the microfluidic chips was mainly based on soft photolithography. First, a mask version of the ITO electrode and polydimethylsiloxane (PDMS) microchannel was designed with CAD 2014. The PDMS microchannel was manufactured as follows. First, the negative photoresist (SU-8 2050) was uniformly poured onto a silicon wafer, spin-coated at 800 rpm for 10 s through a homogenizer, and spin-coated for 30 s at 2500 rpm to produce a 50 *μ*m high PDMS microchannel. After spin-coating, the silicon wafer was baked on a hot plate at 65°C for 2 min and 95°C for 7 min. After baking, the silicon wafer was exposed under 365 nm UV light of the lithography machine for 10 s. The energy density was 12.4 mJ/cm^2^. Then, the silicon wafer was baked with the same parameters on a hot plate. Finally, the wafer was washed twice in the developing solution and dried with nitrogen to obtain a PDMS microchannel mold. Then, 30 g of PDMS and the curing agent were mixed in a weight ratio of 10 : 1. PDMS was poured into the mold, which was then placed in a vacuum oven for 5 min. After baking at 85°C for 30 min, the PDMS microchannels were separated from the mold and cut to the appropriate size. The ITO electrode was manufactured as follows. First, a positive photoresist (RZJ-304) was applied to the ITO conductive glass at 3500 rpm to produce a 2 *μ*m thick photoresist layer. The electrode was baked at 100°C for 3 min and then exposed to 365 nm UV for 2 s at an energy density of 12.4 mJ/cm^2^. After exposure, the electrode was placed in a developer (RZX-3038) for 2 min and blow dried with nitrogen. The exposed ITO conductive glass was then etched away with hydrochloric acid and blown dry with nitrogen to make a patterned electrode. Finally, the PDMS microchannel and ITO electrode were placed in a plasma cleaner for 2 min by oxygen plasma treatment and then baked at 95°C for 15 min to ensure tight bonding. The inlet and outlet of the microfluidic chip were connected to a polytetrafluoroethylene tube.

RETRACTED

### 2.3. Manipulation System

The experimental system for measuring and analyzing the multiangle cellular mechanical properties mainly included the following parts (Figure 2). First, a PDMS-based microfluidic chip was designed and manufactured for the cell stretching experiments. Second, a microfluidic pump (longer pump) was used to inject cells into the microchannels, and then, a signal generator (BK 4014B) was used to generate a sinusoidal voltage waveform. Third, the cell deformation was observed and recorded using a microscope (Nikon) and a CCD camera.

### 2.4. Theoretical Analysis

The DEP force *F*_DEP_ can be estimated by the following formula, in which the red blood cells stretched by DEP were assumed to have an ellipsoid structure [20, 21]:

(1) FDEP=πabcεmRefCM∇Erms2,

where *a* and *b* denote the major and minor radii of the red blood cell, respectively; *c* denotes the thickness of the red blood cell. Radii *a* and *b* were measured by a CCD camera, and *c* was assumed as constant (2 *μ*m) [21]. *f*_CM_ denotes the Clausius–Mossotti factor, *ε*_m_ denotes the permittivity of the suspending medium, Re[*f*_CM_] denotes the actual component of *f*_CM_, and ∇*E*_rms_^2^ denotes the gradient of the square of the applied electric field *E*. The effective permittivity of the red blood cell was estimated with a single-shell structure model as follows [22, 23]:

(2) $$\begin{array}{c} f_{CM}=\frac{1}{3}\frac{\left(\varepsilon_{mem}^{*}-\varepsilon_{m}^{*}\right)\left[\left(\varepsilon_{mem}^{*}+A_{1}\right.\left(\varepsilon_{cyto}^{*}-\varepsilon_{mem}^{*}\right)\right]+\rho \left(\varepsilon_{cyto}^{*}-\varepsilon_{mem}^{*}\right)\left[\left(\varepsilon_{mem}^{*}-A_{1}\left(\varepsilon_{mem}^{*}-\varepsilon_{m}^{*}\right)\right.\right]}{\left(\varepsilon_{m}^{*}+A_{1}\left(\varepsilon_{mem}^{*}-\varepsilon_{m}^{*}\right)\right)\left[\left(\varepsilon_{mem}^{*}+A_{1}\left(\varepsilon_{cyto}^{*}-\varepsilon_{mem}^{*}\right)\right.\right]+\rho A_{2}\left(1-A_{1}\right)\left(\varepsilon_{cyto}^{*}-\varepsilon_{mem}^{*}\right)\left(\varepsilon_{mem}^{*}-\varepsilon_{m}^{*}\right)}, \end{array}$$

where *ω* denotes the angular frequency; *ε* denotes the dielectric permittivity; $j=\sqrt{-1}$; the subscripts cyto, mem, and m represent the cytoplasm, membrane, and medium, respectively; and *ε*^∗^ = *ε* − *jσ*/*ω*. The electrical conductivity is *ρ* = (*a* − *t*)(*b* − *t*)^2^/*ab*^2^, where *t* denotes the thickness of the cell membrane, which was set to 4.5 nm in this study. *ε*_mem_ = 4.44, *ε*_cyto_ = 59, *σ*_mem_ = 10^−6^ S/m, and *σ*_cyto_ = 0.31 S/m [24]. *A*_*i*_ is the depolarization factor which can be given as follows:

(3) $$\begin{array}{c} A_{i}=\frac{1-e_{i}^{2}}{2e_{i}^{3}}\left[\log\frac{1-e_{i}}{1+e_{i}}-2e_{i}\right],\;i=1,2, \end{array}$$

where $e_{1}=\sqrt{1-{\left(b/a\right)}^{2}}$ and $e_{2}=\sqrt{1-{\left(\left(b-2t\right)/\left(a-2t\right)\right)}^{2}}$. The values of Re (*f*_CM_) with the change in the electric field frequency for the red blood cells were calculated by MATLAB R2014a (Figure 3). Therefore, stretching the red blood cell with a frequency of megahertz is more efficient.

RETRACTED

### 2.5. Cell Stretching Protocol

The multiangle stretching of cells could be divided into the following parts. First, the DEP buffer containing red blood cells was passed through the middle microchannel at a flow rate of 5 *μ*l/min, whereas the DEP buffer without red blood cells was passed through the microchannels at both sides at a flow rate of 10 *μ*l/min. This flow rate could concentrate the cells in the middle part of the microchannel and improve the capture efficiency of the cells. Second, a sine wave with a frequency of 1.5 MHz and a peak-to-peak value of 2 Vpp was applied between ITO electrodes 1 and 2. The flow direction of the cells was from right to left (Figure 4(a)). First, ITO electrodes 1 and 2 were connected to increase the probability of capturing red blood cells at the middle edge of ITO electrode 1. The cells were prevented from being caught at the edges of the ITO electrode 2 or 3. When one red blood cell was captured at the edge of the ITO electrode 1, the microflow pump was turned off. The injection of red blood cells and DEP buffer was stopped. Then, the voltage between ITO electrodes 1 and 2 was increased from 2 Vpp to 10 Vpp, and the deformation of the cell between the ITO electrodes 1 and 2 was recorded by a CCD (Figure 4(b)). Second, the voltage applied between ITO electrodes 1 and 2 was turned off. Then, a sine wave signal with a frequency of 1.5 MHz and a peak-to-peak value of 2 Vpp was applied between ITO electrodes 1 and 3. The voltage was increased from 2 Vpp to 10 Vpp. The deformation of the cells in the other direction was recorded by the CCD (Figure 4(c)). Finally, a sine wave signal with the same parameters was applied simultaneously between ITO electrodes 1 and 2 and between ITO electrodes 1 and 3 (Figure 4(d)). Then, the voltage was increased from 2 Vpp to 10 Vpp to record the deformation of the cells in the third direction.

RETRACTED

Figure 5(a) shows the connection between the three ITO electrodes. ITO electrode 1 was connected to ITO electrodes 2 and 3. Figures 5(b)–5(d) illustrate the simulated electric field gradients of the three ITO electrodes under different connection states. When a sine wave with a frequency of 1.5 MHz and a peak-to-peak value of 6 Vpp was applied between ITO electrodes 1 and 2, the direction of the DEP force applied to the cell was deviated to ITO electrode 2 at this time. Similarly, when the same voltage was applied between ITO electrodes 1 and 3, the direction of the DEP force applied to the cells was deviated to ITO electrode 3. When a sine wave with a frequency of 1.5 MHz and a peak-to-peak value of 6 Vpp was simultaneously applied between ITO electrodes 1 and 2 and between ITO electrodes 1 and 3, the cell received a resultant force on the directions of ITO electrodes 2 and 3.

## 3. Results and Discussion

### 3.1. Analysis of ITO Electrode Layout

The width of the ITO electrodes and the distance between them affect the efficiency of cell capture and stretching. Therefore, the arrangement of the ITO electrodes should be specially designed according to the type and size of the cells (Figure 6). In this experiment, the diameter of the red blood cells was approximately 6 *μ*m. Therefore, the width of the ITO electrode was set to 40 *μ*m, which could increase the efficiency of capturing and stretching at the single-cell level. We defined an angle *α* to quantitatively describe the distance between the three ITO electrodes. When *α* > 90°, the distance between ITO electrodes 1 and 2 was too large. When a sine wave with a frequency of 1.5 MHz and a peak-to-peak value of 2 Vpp was applied between ITO electrodes 1 and 2, the cells in the middle of ITO electrode 1 were difficult to capture. By contrast, the cells were more easily captured on the left side of ITO electrode 1, affecting the efficiency of the multiangle stretch measurement of the cells. When *α* < 90°, the cells were easy to capture in the middle of the ITO electrode 1. However, the fabrication of the ITO electrode became more difficult, because the distance between ITO electrodes 2 and 3 was very close. The direction of the DEP force changed slightly, and the effect of the multiangle stretching was not obvious. In summary, we set *α* to 90°, in which the fabrication of the ITO electrodes was relatively simple. When a sine wave with a frequency of 1.5 MHz and a peak-to-peak value of 2 Vpp was applied between ITO electrodes 1 and 2, the cells were easily captured in the middle of the ITO electrode 1. The effect of multiangle stretching on the cells was more obvious.

RETRACTED

The ITO electrode parameters in this experiment are shown in Figure 7. The width of the ITO electrode is 40 *μ*m, the distance between the ITO electrode 2 and the ITO electrode 3 is 40 *μ*m, and the distance between the upper and lower ITO electrodes is also 40 *μ*m.

When *α* = 90°, the electric field at the center and the corners of the ITO electrode 1 is approximately the same, which facilitates capturing cells at the center of the ITO electrode 1. If the cells are not captured in the middle of the ITO electrode 1, the DEP force applied on the cell would be different, which makes it difficult to evaluate the mechanical properties of cells at different angles. When the cell type and size change, it is flexible to adjust the voltage and frequency by using this electrode arrangement. Meanwhile, this electrode form is more convenient for measuring three-angle mechanical properties of cells.

As is shown in Figure 8, the distance between the upper and lower ITO electrodes is 40 *μ*m. When the width of the ITO electrode is 20 *μ*m and 40 *μ*m, the electric field at the center and the corners of the ITO electrode 1 is approximately the same when *α* = 90°, which facilitates capturing cells at the center of the ITO electrode 1. As the width of the ITO electrode 1 is increased to 80 *μ*m, it can be found that the electric field at the corners of the ITO electrode 1 is greater than that of the center. At this time, the distance between the upper and lower electrodes needs to be increased to make *α* = 90°. However, according to the size of the red blood cells (6-8 *μ*m) in this experiment, if the ITO electrode is too wide, many cells may be captured at the edge of the ITO electrode at the same time, and higher voltage is needed to stretch the cells. Therefore, we set *α* to 90°, the width of the ITO electrode to 40 *μ*m, the distance between the ITO electrode 2 and the ITO electrode 3 to 40 *μ*m, and the distance between the upper and lower ITO electrodes to 40 *μ*m.

Figure 9(a) shows the simulation diagram of the electric field gradient in the middle of the ITO electrode 1 at *α* = 90°. The yellow polyline in Figure 9(b) denoted the electric field gradient in the middle of ITO electrode 1 when a sine wave with the same parameters was applied between ITO electrodes 1 and 2 or 3. The magnitude of the electric field gradient at the center of ITO electrode 1 was almost the same because ITO electrodes 2 and 3 were symmetrically arranged at both sides of ITO electrode 1. As the peak-to-peak voltage increased from 1 Vpp to 10 Vpp, the electric field increased from 2.5 × 10^4^ V/m to 2.5 × 10^5^ V/m. The blue polyline in Figure 9(b) denotes the resultant electric field *t* that two sine waves with a frequency of 1.5 MHz were applied between ITO electrodes 1 and 2 and between ITO electrodes 1 and 3. As the peak-to-peak voltage increased from 1 Vpp to 10 Vpp, the resultant electric field increased from 4 × 10^4^ V/m to 3.6 × 10^5^ V/m.

RETRACTED

### 3.2. Cell Stretching Experiments

Figure 10 shows the experimental process of the multiangle stretching of cells. First, a red blood cell was captured in the middle of ITO electrode 1. A sine wave with a frequency of 1.5 MHz was applied between ITO electrodes 1 and 2. Then, the peak-to-peak voltage was gradually increased from 1 Vpp to 10 Vpp. Figures 10(b)–10(d) show the deformation of the red blood cell when the voltage was set to 9 Vpp. As the voltage increased, the DEP force on the red blood cells located in the middle of the ITO electrode 1 also gradually increased. The deformation of the cell along the direction of ITO electrode 2 was recorded by the CCD. Second, a sine wave with the same frequency was applied between ITO electrodes 1 and 3. The voltage between these electrodes was also increased from 1 Vpp to 10 Vpp; the deformation of the cell along the direction of ITO electrode 3 was recorded. Finally, two sine waves with a frequency of 1.5 MHz were applied between ITO electrodes 1 and 2 and between ITO electrodes 1 and 3. The deformation of the cell along the direction of the resultant force was recorded.  Figure 11 shows the change in the DEP force on the red blood cell in the middle of ITO electrode 1 with the increase in voltage. When a sine wave with the same parameters was applied between ITO electrodes 1 and 2 or 3, the cell was subjected to the same DEP force, which was increased from 1 pN to 70 pN. When two sine waves with the same parameters were applied between ITO electrodes 1 and 2 and between ITO electrodes 1 and 3, the resultant force the cell received increased from 2 pN to 136 pN.

The degree of cell deformation was defined as *D* by the following formula:

(4) $$\begin{array}{c} D\left(u\right)=\frac{l\left(u\right)}{l_{0}}, \end{array}$$

where *u* denotes the peak-to-peak voltage of the sine wave, *l*(*u*) denotes the length of the cell after deformation at the voltage of *u*, and *l*_0_ denotes the original length of the cell. As shown in Table 1, the amount of deformation of the cell gradually increased as the voltage was increased from 1 Vpp to 10 Vpp. *D* (*u*1) indicated the deformation of the cell when a voltage was applied between ITO electrodes 1 and 2. *D* (*u*2) indicated the deformation of the cell when a voltage was applied between ITO electrodes 1 and 3. *D* (*u*3) represented the deformation of the cell when all three ITO electrodes were connected. The DEP force in one direction and the resultant DEP force were also included in Table 1 to show intuitively the relationship between cell deformation and DEP force. Analytical results of *D* (*u*1), *D* (*u*2), and *D* (*u*3) show that when the DEP force received by the cell was below 70 pN, the maximum deformation was 1.21. The deformation of the cell in all directions was proportional to the value of the DEP force. Hence, the mechanical properties of the red blood cells were inferred to be almost the same in all directions. Analysis of *D* (*u*3) shows that when the red blood cell was subjected to a DEP force of 100 pN, the deformation reaches a maximum value of 1.38. When the voltage was continuously increased, the DEP force was increased, but the cell deformation did not increase. However, the deformation of the cell continued to increase when the voltage was increased to above 10 Vpp, and this process was irreversible (Figure 12). The cell did not return to its original state after being stretched, and the physiological structure of the red blood cell was destroyed.

RETRACTED

## 4. Conclusions

A microfluidic chip with three unsymmetrical ITO electrodes was innovatively designed to measure and analyze the multiangle cellular mechanical properties. The designed chip had wide practicability, and the measurement and analysis of the multiangle mechanical characteristics of different kinds of cells were achieved by only adjusting the distance between the ITO electrodes. These properties enabled an accurate and comprehensive measurement. An efficient and accurate platform for measuring and analyzing cellular mechanical properties was established. A series of experiments was performed to measure and analyze the multiangle mechanical properties of mouse red blood cells. The results showed that the mechanical properties of red blood cells were almost the same in all directions. This work provides an efficient and low-cost tool for evaluating the multiangle cellular mechanical properties of cells to obtain comprehensive and accurate data. In addition, a new method for generating larger DEP force (resultant force) at low voltages was proposed. This method may increase the efficiency of cell manipulation.

## Figures and Tables

**Figure 1:** Scheme of microfluidic chip. Microfluidic chip consisting of three ITO electrodes and three microchannels.

**Figure 2:** Manipulation system consisting of a signal generator, a microscope, and two microfluidic pumps.

**Figure 3:** Values of Re (*f*_CM_) with electrical frequency between 1 kHz and 100 MHz.

**Figure 4:** Scheme of the cell-stretching process: (a) the microfluidic syringe pump was on, and a sine wave with 2 Vpp and a frequency of 1.5 MHz was applied to capture the red blood cell on the middle of ITO electrode 1; (b–d) injection of DEP buffer was stopped, and the voltage was increased to stretch the cell in different directions.

RETRACTED

**Figure 5:** Simulation of the electric field gradient between the ITO electrodes and the direction of the DEP force.

**Figure 6:** Schematic diagram of the distance between ITO electrodes (scale bar was 20 *μ*m).

**Figure 7:** Diagram of the electric field between ITO electrodes when *α* = 90°.

**Figure 8:** Diagram of the electric field between ITO electrodes. The width of the ITO electrode was set to (a) 20 *μ*m, (b) 40 *μ*m, and (c) 80 *μ*m.

**Figure 9:** (a) Simulation diagram of the electric field in the middle part of ITO electrode 1; (b) diagram of the resultant electric field and the electric field in one direction.

**Figure 10:** Experimental images of cell stretching. (a) A red blood cell was captured in the middle of ITO electrode 1. (b) A sine wave with 9 Vpp and a frequency of 1.5 MHz was applied between ITO electrodes 1 and 2. (c) A sine wave with the same parameters was applied between ITO electrodes 1 and 3. (d) Two same sine waves were applied between ITO electrodes 1 and 2 and between ITO electrodes 1 and 3.

**Figure 11:** Relationship between the DEP force and voltage. The blue line represents the DEP force in one direction, and the red line represents the resultant force.

**Figure 12:** After applying a 10 Vpp sine wave to the ITO electrodes to stretch the cell, the cell did not return to its original shape. The scale bar was 20 *μ*m.

**Table 1:** DEP force and cell deformation.

Voltage (Vpp)	DEP force in one direction (pN)	*D* (*u*1)	*D* (*u*2)	Resultant DEP force (pN)	*D* (*u*3)
1	1	1.0	1.0	2	1.0
2	3	1.02	1.02	6	1.03
3	6	1.04	1.03	12	1.07
4	10	1.05	1.06	20	1.11
5	16	1.10	1.10	36	1.15
6	24	1.13	1.13	48	1.17
7	32	1.15	1.14	68	1.20
8	42	1.16	1.15	88	1.25
9	56	1.19	1.18	108	1.38
10	70	1.21	1.21	136	1.38

## Data Availability

All the data underlying the finding of this study can be accessed by emailing the corresponding author Hao Yang (yhao@suda.edu.cn).
